# Analysis of the Impact Mechanism of Occupational Identity on Occupational Well-Being Based on Big Data

**DOI:** 10.1155/2022/4870296

**Published:** 2022-05-29

**Authors:** Yuefen Wang, Dianyi Yang

**Affiliations:** School of Marxism, Northeast Forestry University, Harbin 150040, China

## Abstract

Occupational identity is an individual's view, recognition, and approval of his long-term occupation, and its importance to every professional is self-evident. Only when a professional person agrees with the profession he is engaged in from the bottom of his heart can he devote himself wholeheartedly to it and unreservedly exert his greatest potential. On the basis of sorting out and analyzing the prevailing theoretical and empirical research results, this paper deliberates the empirical research on the influence mechanism between employees' occupational identity and occupational well-being. In this study, through big data analysis, literature search, questionnaire survey, and other methods, this paper obtained the professional identity data of employees in different companies and used a method of big data analysis, namely, BP neural network (BPNN) to design in this paper to verify the data, and finally obtain an effective theoretical model of the influence mechanism of occupational identity and occupational well-being. The main work of this paper is as follows: (1) it introduces the interpretation of the concept of “professional identity” by different scholars at home and abroad and makes a brief review of the researches on professional identity and professional well-being made by foreign scholars in recent years. (2) The basic knowledge and algorithm process of artificial neural network (ANN) are introduced, and the design of the evaluation model of the influence mechanism of occupational identity on occupational well-being based on BPNN is proposed. (3) The simulation software validates the neural network (NN) assessment system developed in this paper. Experiments reveal that the BPNN system is a reasonable and feasible evaluation approach for analyzing the impact of occupational identity on occupational well-being.

## 1. Introduction

Identity is generally believed to be derived from psychology. The famous psychologist Freud believed that identity is a process of human cognition and is the inner emotional connection between individuals and individuals, individuals and groups, and individuals and society. The individual's attitude towards the identification of the external world is embodied in the orientation of values [1–3]. An individual's sense of identity is a continuous process that will be precious by the surrounding environment. Once formed and transformed into a part of one's own cognition, it is difficult to change. Identity is the internal acceptance of the object by the subject, and it shows consistency in values and behaviors. Occupational identity is an individual's value orientation towards a certain occupation, with an attitude of approval, affirmation, and yearning. This occupational role attracts the individual's attention and conforms to emotional experience, and the individual will strive to become a part of this type of occupation [4–6]. Occupational identity is a continuous dynamic process, and occupational identity has the same root and origin as “self-identity” in psychology. High occupational identity has a promoting consequence on individual work and can help individuals to do their job well. Occupational identity is embodied in many aspects and is an important criterion for measuring individual occupational mental health. Reference [7] believes that one of the internal factors affecting happiness is employees' professional identity. Nowadays, “happiness” is what employees of every enterprise want to pursue, and enterprise managers should also skillfully use the theory of happiness in the process of management according to the situation. Whether employees are happy or not will have a great impact on an enterprise. If an employee feels that he is very happy in this enterprise, then, he will preserve a loyal attitude towards the enterprise, be full of energy at work, and there will be a respectable relationship between the employee and the enterprise. Labor relations and job performance are correspondingly higher, and vice versa [8]. If this condition continues for a long time, the enterprise will have such a condition: the market competitiveness will gain absolute advantage and will preserve the momentum of development. As a manager of an enterprise, you should clearly know that money is not what people really want, because even if you have money, it is for a good and happy life, and money serves life, so managers must understand that his employees ultimately what I want to pursue is “happiness” itself. This requires that enterprise managers should master the corresponding psychological knowledge, use the theory of happiness, and carry out scientific and reasonable management and decision-making under limited resources, so that employees can work and be happy. Based on the above analysis, it is necessary to study the influence mechanism of employees' occupational identity on their subjective well-being. Whether an employee of an enterprise agrees with his occupation and the degree of identity will directly affect his work progress and quality of life, and then, it is related to the organizational efficiency of the enterprise and the realization of the ultimate goal. Since NN is also an important method of data mining, it has excellent processing ability for nonlinear problems.

This paper focuses on using BPNN to study the influence mechanism of occupational identity on subjective well-being. The centripetal dimension refers to teachers' awareness of the importance of their professional identity in their work. Therefore, this study adopts the method of data mining to analyze the influence mechanism of employees' occupational identity on their subjective well-being.

## 2. Related Work

Identity is a concept closely related to the study of various academic circles, such as social identity, cultural identity, national identity, and political identity. Among them, social identity refers to the convergence of individual behaviors, values, and social norms, and one of its manifestations is occupational identity. Reference [9] first started from the perspective of identity theory and pointed out that occupational identity is the stability and clarity of an individual's understanding of the goals, values, and meanings of occupations, but they emphasize that occupational identity is a relatively stable state. Subsequently, reference [10] pointed out that occupational identity is a concept that is gradually constructed and matured in the process of psychological development and will change with continuous social learning and interaction. Reference [11] defines it from the perspective of the form adopted by professional identity. It believes that professional identity is an unconscious whole in the form of gestalt about needs, goals, emotions, values, prior knowledge, and behavioral inclinations. This will in turn affect professional beliefs and behavioral aspects. Reference [12] pointed out that occupational identity is the evaluation of one's own ability and the thinking and clarification of occupational values in the process of engaging in occupation. To sum up, professional identity is not only an instrumental role played in the professional background nor is it a simple synthesis of a professional's achievements, values, and beliefs. We can think of occupational identity as an individual's cognition and construction of a specific occupation and self-role concept gradually developed from growth experience and social interaction. Reference [13] pointed out that teachers' professional identity is no single or absolute nor can it be static and immutable. It is a dynamic process that requires multifaceted, multiangle, and multilevel research and analysis. In the process of identification, teachers are constantly accumulating experience and constantly criticizing and correcting. Reference [14] proposes that the professional image of teachers reflects the professional role of employees to a large extent, which is relatively complex and a dynamic process. The formation process of employees' occupational roles is the formation process of occupational identity. Reference [15] introduced the individual's perception of occupation, such as entry motivation, working conditions, and life choices, into the category of teachers' occupational identity. Through the research on occupational identity, occupational identity is divided into four dimensions, namely, the level of centrality, the level of value, the level of solidarity, and the level of self-expression. The value dimension indicates that employees identify with their occupational value, and the occupation is more attractive. The solidarity dimension indicates that employees value the group and focus on good interpersonal relationships with colleagues. Employees can be appreciated, acknowledged, and loved by society, the company, colleagues, and others, and give greater attention to their own emotional attitudes, thanks to the dimension of self-expression. Reference [16] pointed out that in the research on the formation of employees' professional identity, the interaction between the individual and the collective is very important. Reference [17] conducted research on teachers' professional identity and came to a conclusion, starting from three aspects including emotion, persistence, and norm. Reference [18] believes that employees' professional identity has a great correlation with professional reality cognition. Reference [3] concluded through case studies that individual reflection helps professional identity development. Reference [19] found through research that occupational identity and turnover intention were significantly negatively correlated, occupational identity was closely related to turnover intention, and the level of occupational identity was poor, then turnover intention was relatively high. As domestic and foreign scholars gradually deepen their research on the internal aspects of the company's employees, they have made great progress in the professional identity of employees. My country mainly conducts quantitative research in this area, and the content of the research is mainly reflected in the analysis of the status quo of employees' occupational identity and the research on its relationship with other aspects. Because occupational identity and organizational identity are based on social identity theory, they are both developed on the basis of social identity theory. Therefore, as far as the current foreign professional identification assessment tools are concerned, most of them are formed after the adaptation of the organizational identification assessment tools. This paper chooses a more representative scale, “Professional Identification Scale.” The occupational identity scale developed by Brown et al. was initially composed of three dimensions: awareness of occupational membership, positive evaluation of occupational groups, and sense of belonging to occupational groups. After multiple structural validity tests, a single-dimensional scale was formed, consisting of 10 items, and scored on a Likert 5-point scale. The stronger the professional identification, the higher the score. The Cronbach's alpha coefficient of this scale is 0.71, which is a relatively widely used measurement tool at home and abroad. The Chinese version of the single-dimensional structure scale has a Cronbach's alpha coefficient of 0.82, and its reliability and validity are also relatively good.

Because most international researchers feel that work is a significant aspect of life, it should be included in studies of professional well-being [20]. Researchers disagree on the idea and structure of occupational well-being, according to a study of international literature. Reference [21], for example, suggested a two-dimensional model of emotion, health, and behavior based on the assumption that health is an important indication of well-being, in which behavior corresponds to work ability and ambition and placed job potential under the health dimension. The concept of health was integrated into one dimension, causing confusion. Reference [2] put forward a five-dimensional model of occupational well-being on the basis of synthesizing the results of previous researches, arguing that occupational well-being is an individual's evaluation of various aspects of their work, including cognitive, emotional factors, personal development, physical, and mental health and behavior. Therefore, to sum up, although the opinions of various researchers are inconsistent, they all emphasize that the measurement of occupational well-being should be based on the perspective of development, focusing on the background of well-being. In recent years, occupational well-being has gradually become the focus of domestic researchers. Some researchers believe that occupational well-being is the happiness experience of professionals in occupational activities, and it is the reflection of subjective well-being in the workplace, including emotional experience and recognition. There are two dimensions of knowledge evaluation, but there is no exact definition of the concept of occupational well-being [22]. Reference [23, 24] believes that occupational well-being is a relatively stable emotional experience dominated by positive emotions, which is accompanied by an individual's judgment of his or her occupational identity, occupational activity process, and occupational benefits and focuses on the satisfaction of spiritual needs and positive emotions, so professional well-being places more emphasis on the spiritual dimension of self-realization. We can know that occupational well-being is a multidimensional and flexible concept, and it is also a key indicator of an individual's comprehensive evaluation of occupation. Therefore, a broader concept of well-being can help recover the well-being of professional people and formulate relatively broad intervention strategies. In this sense, a broad conceptualization enriches the theory and practice of occupational psychology.

## 3. Method

### 3.1. Artificial Neural Networks

In the evaluation of nonlinear problems, traditional common methods have many defects. ANNs can learn and train from a large amount of complex data with unknown patterns and find their regularity, especially, they can process any type of data. This is not possible with traditional methods. Therefore, applying the theory of ANN to analyze the influence mechanism of occupational identity on occupational well-being not only overcomes the problems of establishing complex mathematical analytical expressions and mathematical models in the traditional evaluation process but also avoids artificial subjective randomness. It is an effective way to evaluate the mechanism. NNs can be divided into biological NNs and ANNs. All of the NNs mentioned in this article are ANNs. NNs are a typical method to realize artificial intelligence through physiological structure simulation. It starts from the physiological structure of the human brain. Using the point of view of bionics to explore the mechanism of human intelligent activities, it is a method that combines the research on the microstructure of the human brain with the research on intelligent behavior. NN systems are highly nonlinear and self-adaptive and are often used to simulate intelligent behaviors such as cognition, decision-making, and control. The research of NN theory has laid the foundation for people to solve the parallel processing and parallel computing problems of large-scale information processing. Since the 1980s, NN theory has entered a period of rapid development, which has attracted the attention of scholars in many fields and penetrated into all engineering application fields. So far, NN has become a frontier research topic that has developed rapidly in the world.

Synaptic connections in the brain are used to process information in this mathematical model of ANN. Signals are routed across the system through processing units and channels. In addition to having local memory, these processing units may also perform local operations. There are multiple parallel connections for each processing unit, but the one-to-one output remains constant regardless of how many parallel connections are used; this means that even if the number of parallel connections is increased or decreased, each processing unit's signal and its magnitude remain constant. Any mathematical model may be used as the processing unit's output signal, and each processing unit performs local operations. The processing unit must only be constructed on the value stored in the local scope of the processing unit and the existing value of all input signals that influence the processing unit over the input. There are a vast number of nodes and interconnections between them in the NN, which is a model of functioning. The excitation function denotes the output function implied by each node. The memory of an ANN is represented by the weight of each link between two nodes, which is referred to as a weight. The output of the network is dependent on the weight of the network, the technique of connection, and the excitation function. Each individual neuron in the brain is connected to the rest of the network through connections called neurons. There are various learning algorithms for NNs.

#### 3.1.1. Hebb Type Learning

The idea of Hebb-type learning has a certain biological background, and its idea can be summarized into two points: if two neurons on both sides of a synapse are activated at the same time, the energy of the synapse will be selectively increased; conversely, if two neurons on either side of a synapse are activated asynchronously, the synapse's energy is selectively reduced. The mathematical description is as follows:

(1) $$\begin{array}{c} ∆w_{ij}\left(n\right)=\varepsilon \left(x_{j}\left(n\right)-{\bar{x}}_{J})(x_{i}\left(n\right)-{\bar{x}}_{I}\right). \end{array}$$

#### 3.1.2. Error Correction Type Learning

Error correction learning is a supervised learning process. The reference basis for adjusting the connection weights is the deviation between the expected output of the NN and the actual output and ultimately reduces this deviation.

#### 3.1.3. Random Learning

The random learning algorithm introduces methods such as random process and probability into the algorithm, adjusts the variables of the network through these methods, and further maximizes the objective function of the network.

#### 3.1.4. Competitive Learning

Competitive learning is to introduce a competitive mechanism into the learning algorithm. All units in a certain part of the NN compete to obtain who is the output. The unit connection weight that wins in the competition changes to a more favorable direction for the competition of this input stimulus pattern. Furthermore, the winning unit inhibits the response of the losing unit to the stimulus pattern, so that only one output neuron is active at any one time.

#### 3.1.5. Learning Based on Memory

Memory-based learning is mainly used for pattern classification, such as nearest neighbor classifiers.

#### 3.1.6. Structural Revision Learning

The modification of the NN structure, that is, the change of the network topology, also plays an important role in the learning process of animals. That is to say, the learning of the NN is not only reflected in the changes of the weights but also the changes of the network results will also affect the learning.

### 3.2. BP Neural Network

The multilayer feed-forward NN has greatly improved the classification ability of the network due to the introduction of the hidden layer. Since the error back-propagation method is often used in the training of the multilayer feed-forward network, the multilayer feed-forward network is often called BPNN.

#### 3.2.1. BP Algorithm Model

Forward propagation and backward propagation of the mistake are two separate processes in BP's learning process. Forward propagation shows that input samples are first received from an external source, then managed by each hidden layer, and then sent to a final output layer. Errors will be propagated backward if there is a significant difference between the actual output of the output layer and what was intended. Errors are propagated backwards in a layer-by-by-layer fashion from the output layer to the hidden layer and finally to the output layer via back-propagation error correction. Back-propagation distributes the mistake to each layer's units, and the apportionment results for each layer. As a foundation for the error signal, the weight of each unit and its error signal is rectified. The two sections of the BP algorithm cycle repeatedly to alter the weights of each layer in the learning process. The weights of each layer of the network are constantly being adjusted throughout the network's learning and training phase. Until the network output error is within an acceptable range or the number of loops hits the top limit, the two sections are looped back and forth.

#### 3.2.2. BP Learning Algorithm

Figure 1 depicts the most generally used NN, as well as the most popular single hidden layer NN. The input layer, the hidden layer, and the output layer are the three layers of this single hidden layer feedforward network, which is also known as a three-layer perceptron or a three-layer feedforward network.

The fundamental of the BP algorithm is to iteratively obtain the minimum error value. The error *E* between the network output and the expected output is as follows.

(2) $$\begin{array}{c} E=\frac{1}{2{\left(b-O\right)}^{2}}=\frac{1}{2\sum_{k=1}^{1}{\left(b_{k}-O_{k}\right)}^{2}}. \end{array}$$

The formula of the error *E* in the hidden layer is as follows:

(3) $$\begin{array}{c} E=\frac{1}{2}\overset{1}{\underset{k=1}{\sum }}{\left[b_{k}-g\left(\overset{m}{\underset{j=0}{\sum }}w_{jk}y_{j}\right)\right]}^{2}. \end{array}$$

The formula for the error *E* in the expansion to the output layer is as follows:

(4) $$\begin{array}{c} E=\frac{1}{2}\overset{1}{\underset{k=1}{\sum }}{\left\{b_{k}-g\left[\overset{m}{\underset{j=0}{\sum }}w_{jk}g\left(\overset{n}{\underset{i=0}{\sum }}V_{ij}x_{i}\right)\right]\right\}}^{2}. \end{array}$$

From formula (4), the input error of the BPNN is also the weight function of the overall layers, and the change of the error can be achieved by adjusting the weights. Using gradient descent, the weights are continuously adjusted as follows.

(5) $$\begin{array}{c} \Delta w_{jk}=-\frac{\lambda \partial E}{\partial w_{jk}},j=0,1,\cdots ,m;k=1,2,\cdots ,l. \end{array}$$

(6) $$\begin{array}{c} \Delta V_{ij}=-\frac{\lambda \partial E}{\partial V_{ij}},i=0,1,\cdots ,n;j=1,2,\cdots ,m. \end{array}$$

After repeated cycles, the value adjustment function of the weight of the BP learning algorithm is

(7) $$\begin{array}{c} \Delta w_{jk}=\lambda \theta_{k}^{O}y_{j}=\lambda \left(b_{k}-O_{k}\right)O_{k}\left(1-O_{k}\right)y_{j}, \end{array}$$

(8) $$\begin{array}{c} \Delta V_{ij}=\lambda \theta_{j}^{y}x_{i}=\lambda \left(\overset{l}{\underset{k=1}{\sum }}\mu_{k}^{O}w_{jk}\right)y_{j}\left(1-y_{j}\right)x_{i}. \end{array}$$

In the BP learning algorithm, the weight adjustment formula of each layer of the network is the same in form, and the formula is determined by three factors, namely, the output error signal *θ* of this layer, the learning rate *λ*, and the input signal *X* (or *Y*). The error signal of the output layer comes from the transformation of the difference between the expected output and the actual output. The error signal of each hidden layer depends on the error signals of the layers before the layer. These error signals are all back-transmitted from the output layer by layer.

#### 3.2.3. Defects of BP Algorithm

The BP algorithm can estimate any nonlinear function with any precision after being used in a three-layer feedforward network with a nonlinear transfer function, which is the reason why the BP network is more and more widely used. However, the standard BP algorithm has some inherent defects in its application:

1. It is easy to not obtain the global optimal solution and only obtain the local minimum solution
2. Too many training times will reduce the learning efficiency and slow down the speed of convergence
3. The selection of hidden nodes lacks theoretical guidance
4. During training, learn new samples but easily forget about old samples

#### 3.2.4. Improvement of BP Algorithm

In order to overcome the shortcomings of the BP algorithm, a variety of new algorithms have been proposed to improve it in practice, and the network has been improved from different angles.

1. Simulated annealing algorithm

It is a global optimization algorithm that simulates the metal annealing process. The adjustable weights of the network are equivalent to the particles in the metal, and the output error of the network is equivalent to the energy state of the metal. By adding “noise” to the variables, it is possible for the network to jump out of the minimum point of the cost function and converge to the global minimum point.

(2) Genetic algorithm

It is a probabilistic search method that mimics the genetic and evolutionary processes of animals in the wild. It is an adaptable global optimization algorithm. A number of beginning points are used to avoid the network from settling on a local solution instead of a global one; the algorithm employs the probability law to guide its search and conducts efficient heuristic search in the solution space. We would prefer thorough yet methodical research than haphazard or unfocused efforts. As a result, avoiding local minima is extremely probable. Apply the global search performance of a genetic algorithm first, and then use error back propagation to identify a solution that is best for your particular situation.

(3) Improve the normalization algorithm of training samples

Due to the large difference in the physical quantities of the input nodes of the network, the training samples of various indicators are not comparable, so the evaluation cannot be carried out smoothly. In order to prevent small values from being overwhelmed by large values, different normalization methods can be used to normalize the input samples to between [0, 1].

(4) Reasonable selection of initial weights and thresholds

By selecting appropriate weights and thresholds, or making appropriate adjustments during the training process, the global optimal solution can be achieved to jump out of the local minimum area. In many literatures, a variety of initial values are set, and then, the one with the best training effect is selected as the weight and threshold after learning. This method is relatively simple and effective and is widely used.

(5) Improve the activation function

In the hidden layer of the network, the activation function of neurons generally uses the *S* function, but the *S* function has a defect. When the value is close to 0 or 1, the regions at both ends are defined as the saturated region, and the middle region is the unsaturated region. In the saturation region, the change of the independent variable has been unable to change the change of the function value well. If the output of the network neuron is different from the expected value at this time, and the adjustment amount of the connection weight is small, it is difficult to adjust the existing state of the neuron, and the convergence speed is slowed down, which is the “platform” phenomenon. In order to solve this problem, the activation function of the neurons in the hidden layer can be in the form of formula (9). By adjusting the values of *d*, *g*, and *h*, the saturation region of the function can be changed, so as to attain the determination of adjusting the output value of the neuron.

(9) $$\begin{array}{c} f\left(x\right)=\frac{1}{d}+ge^{-hx}. \end{array}$$

(6) Adjust the network structure

The network structure is changed by increasing the number of nodes, layers, and connection methods according to certain rules, so as to solve the problem that the global optimal solution and the local minimum cannot be obtained.

(7) Determination of the number

Determination of the number of neurons in the hidden layer if the level of the network is certain, the increase in the number of hidden layers can effectively improve the training accuracy. The premise of ensuring that a nonlinear network has the ability to approximate any curve is to have enough hidden layer neurons, but if there are too many hidden layer neurons, the convergence speed will be slowed down. There is a theory in the literature that if there is a node in the input layer of a three-layer feedforward NN, then when the number of nodes in the hidden layer is 2*a* + 1, the network can approximate any differentiable function with arbitrary precision.

### 3.3. Evaluation Index System Based on BPNN

The index system plays a critical role in the evaluation of nonlinear problems since it is scientific and fair. In the index system, the meaning and weight of each index are marked in detail, and the reasonable and scientific settings of the index system play a key role in the evaluation system. Regardless of the final result of the evaluation or the evaluation index of the evaluation index system, the correspondence between the rank and the output range is shown in Table 1. The evaluation system proposed in this paper for the impact of occupational identity on occupational well-being is designed with multiple evaluation indicators, as shown in Table 2.

### 3.4. Evaluation Data Initialization Processing

Since the input of indicators in this article is obtained by scoring or grades, the percentage system is used. However, the input data range of the BPNN is between [0, 1], and the excitation function is the *S* function. Therefore, before the NN is trained, the input data should be normalized. Commonly used normalization functions are the maximum and minimum method, exponential function method, and so on. This paper uses the maximum and minimum method to normalize the input data. This method is a linear transformation of the data, which can better preserve the original meaning of the data. The input data normalization formula is as follows:

(10) $$\begin{array}{c} X=I-\frac{I_{\min}}{I_{\max}}-I, \end{array}$$

where *X* is the input value of the BPNN, *I* is the evaluation original data, *I*_min_ is the minimum value of the BPNN input, and *I*_max_ is the maximum value of the BPNN input.

## 4. Experiment and Analysis

### 4.1. Determination of BP Network Results

According to Kolmogorov's theorem, a BPNN with a hidden layer can be used to approximate any continuous function mapping relationship. Any continuous rational function in a closed interval can be approximated by a BPNN with a sigmoid hidden layer and a linear output layer. Therefore, in the design of BPNN, the three-layer network can meet the basic requirements. If the number of layers is enlarged, the complexity of the network will be greatly enlarged, the training time will be increased, and the scope of reducing the error will be limited. This paper constructs the evaluation model using the three-layer BP network structure.

1. The number of neural units in the input layer is determined

The number of neural units in the input layer is determined as the number of indicators in the evaluation table, and the available indicators are 10, that is, the number of neural units in the input layer of the BPNN is 10.

(2) The number of neural units in the output layer is determined

The number of neural units in the output layer is the evaluation result of the influence of occupational identity on occupational well-being, which is set to 1 in this paper. Through the qualitative and quantitative evaluation analysis of the course, a quantitative evaluation result output is finally obtained.

(3) The number of neurons in the hidden layer is determined

In the BPNN, the number of neurons in the hidden layer has a great influence on the performance of the NN. If the number of neurons in the hidden layer is too small, the learning ability of the NN will be insufficient, and the network will easily fall into a local minimum point. Sometimes even unstable results may be obtained. On the contrary, if the number of NN elements in the hidden layer is too large, the network will fit the irregular information existing in the sample, resulting in the phenomenon of “overfitting” in the network, which will not only lead to prolonged training time but also errors are not necessarily minimal. Therefore, the appropriate selection of the number of neurons is a very important task. According to experience, for a three-layer NN, the following formula is used for the number of neural units in the hidden layer:

(11) $$\begin{array}{c} h=\sqrt{i+k}+c, \end{array}$$

where *i* is the number of neurons in the input layer, *k* is the number of neurons in the output layer, and *c* is a constant in the range [1–10].

According to the above empirical formula, the number of neurons in the hidden layer of the network model in this paper ranges from [4–14], and the most suitable number of neurons needs to be verified through experiments. The experimental results obtained are shown in Figures 2–4. Finally, 8 is the number of neurons in the hidden layer.

(4) Determination of the training function

Different training functions have different convergence accuracy and number of training steps. From the experimental data, it is most appropriate to choose LM as the training function in this paper.

(5) Determination of the learning rate

In the BPNN, the learning rate remains unchanged. If the learning rate is too large, the network weights will be adjusted to a larger extent each time they are updated, which may cause the NN to jump back and forth around the minimum error value during the update iteration process. When it is true, the network diverges and cannot converge. On the contrary, if the learning rate is too small, the adjustment speed of the network weights will be small each time, and the convergence speed will be slow. Taken together, although the learning rate is small, the convergence rate will be slow, but it will eventually converge to the vicinity of the minimum error value. Therefore, this paper tends to choose a smaller learning plastic sheet to ensure the stability of the system, and the learning rate finally determined in this paper is 0.025.

(6) Determination of activation function

In this paper, the tagsig hyperbolic tangent function is used as the activation function on the hidden layer unit. As mentioned above, the BPNN evaluation system in this paper performs data normalization processing in the first step, so the activation function of the output layer unit is selected as the sigmoid function.

### 4.2. Data Sources

The experiments in this paper are based on the MATLAB software package launched by MathWorks for modeling. This software package is not only a very practical and effective scientific research programming software environment but also an interactive program for scientific nuclear engineering calculation. MATLAB NN toolbox is the activation function of several typical NNs based on the theory of this algorithm designed by using scripting language and provides the function calling method, which is convenient for users to directly call the activation function of the network without repeated construction. Users can also alter the weights according to the specific conditions of the network they developed, as well as the network's training process, write design and training functions suitable for their own network using the scripting language, and learn the functions. At present, the MATLAB NN toolbox contains most of the NNs, including the perceptron model, the BPNN, and the self-organizing network model. In this paper, the results of 280 occupational identity scale B of employees in different types of companies are obtained through online questionnaire survey as experimental data. The screening of the survey data is to delete 5% of the lowest and highest scores to prevent “spam.”. After that, the experimental data is initialized, and the following 240 data are randomly selected as training and simulation data.

### 4.3. Experimental Results of BPNN Model

Through model initialization, a network prediction model is created, and after training the NN, the obtained model is subjected to data-based simulation tests, and the final experimental results are shown in Table 3.

As shown in Table 3, the evaluation results after network training are compared with the actual evaluation results, in which the actual evaluation results are the evaluation data given by experts. From the experimental data, it can be concluded that the training accuracy of the evaluation model of the influence mechanism of occupational identity on occupational well-being based on BPNN is completely acceptable, and it is a scientific, reasonable, and feasible prediction model.

## 5. Conclusion

Wages, bonuses, benefits, and working circumstances, according to motivation theory, are external motivating factors for a person's work motivation, whereas belonging, respect, achievement, and challenge are internal motivational factors for a person's work motivation. Occupational identity is an individual's affirmative evaluation of the occupation he is engaged in. It not only overcomes the externality and sense of alienation of the occupation but also is a person who can internally unify his personal value and meaning with the value and meaning of the occupation he is engaged in. As a result, the occupational work motivation formed on the basis of occupational identity is more conscious, active, and active. Compared with various other external stimuli and inducements, occupational identity plays a more lasting and stable role. In addition, the final experimental results of this paper show that occupational identity has a positive effect on employees' occupational well-being, which can allow employees to bring greater benefits to the enterprise. Therefore, enterprise managers can take the cultivation of employees' professional identity as part of the enterprise culture. The work completed in this paper is as follows: (1) it introduces the interpretation of the concept of “professional identity” by different scholars at home and abroad and makes a brief review of the research on professional identity and professional well-being made by foreign scholars in recent years. (2) The basic knowledge and algorithm flow of ANN are introduced, and the evaluation model based on BPNN is proposed, including NN evaluation model, network structure, learning parameters, and learning algorithm. (3) The NN evaluation system constructed in this paper is verified by the simulation software. Experiments reveal that the BPNN system proposed in this study is a reasonable and feasible evaluation model for determining the process by which occupational identity influences occupational well-being.

## Figures and Tables

**Figure 1:** A single hidden layer NN structure.

**Figure 2:** Train effect when *N* = 4 and *N* = 6.

**Figure 3:** Train effect when *N* = 8 and *N* = 10.

**Figure 4:** Train effect when *N* = 12 and *N* = 14.

**Table 1:** NN output value and evaluation level corresponding table.

Evaluation level	NN output value
Totally suitable	0.900-1
Basically meet	0.800-0.890
Uncertain	0.700-0.790
Basically does not meet	0.600-0.690
Totally inconsistent	0-0.590

**Table 2:** Occupational identity scale assessment indicators.

Index	Label
Work matches my expectations	X1
Work makes me proud	X2
Very satisfied with the work	X3
If you choose a job again, you will still choose the current one	X4
I want my children to do my current job	X5
I would like to do this job for the rest of my life	X6
Your current job is an important part of your self-image	X7
I really identify with my work	X8
The work I do will make me feel more fulfilled than others	X9
My career trajectory is important to realizing my self-worth	X10

**Table 3:** Statistics of the final experimental results.

Result type	Num						
	1	2	3	4	5	6	7
Network evaluation results	0.829	0.815	0.728	0.925	0.682	0.871	0.966
Actual evaluation results	0.827	0.814	0.735	0.919	0.685	0.867	0.970
Error	0.020	0.010	0.070	0.060	0.030	0.040	0.040

## Data Availability

The datasets used during the current study are available from the corresponding author on reasonable request.
